The article "Analysis of the Molecular Mechanism of Evodia rutaecarpa Fruit in the Treatment of Nasopharyngeal Carcinoma Using Network Pharmacology and Molecular Docking" was retracted in 2023. Reasons: suspected computer-generated content; unreliable results or conclusions; concerns about the data; concerns about the results or conclusions.

# Analysis of the Molecular Mechanism of *Evodia rutaecarpa* Fruit in the Treatment of Nasopharyngeal Carcinoma Using Network Pharmacology and Molecular Docking

**DOI:** 10.1155/2022/6277139

**Published:** 2022-04-13

**Authors:** Runshi Xu, Ximing Yang, Yangyang Tao, Wang Luo, Yu Xiong, Lan He, Fangliang Zhou, Yingchun He

**Affiliations:** ^1^Hunan University of Chinese Medicine, Hanpu Science and Education Park, Changsha, China; ^2^First Affiliated Hospital, Hunan University of Chinese Medicine, Changsha, China; ^3^Hunan Engineering Technology Research Center for Prevention & Treatment of Ophthalmology and Otolaryngology Diseases and Visual Function Protection with Chinese Medicine, Hunan University of Chinese Medicine, Changsha, China; ^4^Hunan Key Laboratory for Prevention & Treatment of Ophthalmology and Otolaryngology Diseases with Chinese Medicine, Hunan University of Chinese Medicine, Changsha, China

## Abstract

**Background:**

Nasopharyngeal carcinoma (NPC), a neoplasm of the head and neck, has high incidence and mortality rates in East and Southeast Asia. *Evodia rutaecarpa* is a tree native to Korea and China, and its fruit (hereafter referred to as Evodia) exhibits remarkable antitumour properties. However, little is known about its mechanism of action in NPC. In this study, we employed network pharmacology to identify targets of active Evodia compounds in nasopharyngeal carcinoma and generate an interaction network.

**Methods:**

The active ingredients of Evodia and targets in NPC were obtained from multiple databases, and an interaction network was constructed via the Cytoscape and STRING databases. The key biological processes and signalling pathways were predicted using Gene Ontology and Kyoto Encyclopaedia of Genes and Genomes pathway enrichment analyses. Molecular docking technology was used to identify the affinity and activity of target genes, and The Cancer Genome Atlas and Human Protein Atlas databases were used to analyse differential expression. Cell Counting Kit-8 (CCK-8) and Annexin V-fluorescein isothiocyanate (FITC)/propidium iodide (PI) dual-fluorescence staining were used for experimental verification.

**Results:**

Active Evodia compounds included quercetin, isorhamnetin, and evodiamine, and important NPC targets included MAPK14, AKT1, RELA, MAPK1, JUN, and p53, which were enriched in lipid and atherosclerosis signalling pathways. Additionally, we verified the high affinity and activity of the active compounds through molecular docking, and the target proteins were verified using immunohistochemistry and differential expression analyses. Furthermore, CCK-8 assays and Annexin V-FITC/PI dual-fluorescence staining showed that isorhamnetin inhibited the proliferation of NPC cells and induced apoptosis.

The article "Analysis of the Molecular Mechanism of Evodia rutaecarpa Fruit in the Treatment of Nasopharyngeal Carcinoma Using Network Pharmacology and Molecular Docking" was retracted in 2023. Reasons: suspected computer-generated content; unreliable results or conclusions; concerns about the data; concerns about the results or conclusions.

**Conclusion:**

Our results identified the molecular mechanisms of Evodia and demonstrated its ability to alter the proliferation and apoptosis of NPC cells through multiple targets and pathways, thereby providing evidence for the clinical application of Evodia.

## 1. Introduction

Nasopharyngeal carcinoma (NPC) is an Epstein–Barr virus (EBV) associated epithelial head and neck neoplasm, with the highest incidence and mortality rates occurring in East and Southeast Asia and a 5-year survival rate of only approximately 50% for patients with advanced disease [1, 2]. NPC is highly malignant, has a high recurrence rate, is prone to distant metastasis, and occurs as an advanced disease in more than 50% of patients at diagnosis [3]. NPC is a major public health problem in many countries, particularly in Southeast Asia and North Africa, and its aetiology is considered to be related to various risk factors, such as a family history of the disease, diet containing high-risk ingredients (such as large amounts of nitrosamine compounds and volatile nitrosamines), and previous EBV infection [4, 5]. Comprehensive treatment with conventional conformal radiotherapy and cisplatin-based adjuvant chemotherapy is the preferred regimen for treating NPC [6]; however, disease recurrence and distant metastasis are the main factors associated with treatment failure. Such a treatment regimen can also result in concurrent and severe adverse reactions; therefore, the development of a new model for treating NPC is critical.

The use of traditional Chinese medicine (TCM) to treat NPC is attaching increasing attention. TCM has fewer side effects and adverse reactions than Western chemotherapeutic drugs and presents a lower risk of patients developing drug resistance. Evodia (*Tetradium ruticarpum* (A.Juss.) T.G.Hartley (Rutaceae)) is the dry and nearly mature fruit of rutaceous plants (*Evodia rutaecarpa* (Juss.) Benth. var. Officinalis (Dode) Huang or *E. rutaecarpa* (Juss.) Benth. var. bodinieri (Dode) Huang). Recent studies have shown that the main Evodia compounds are alkaloids, bitterin, volatile oil, and flavonoids, among which quercetin, evodiamine, and isorhamnetin are the main active compounds [7–9]. A pharmacological study indicated that Evodia has analgesic, anti-inflammatory, anti-ulcer, and anti-tumour effects in addition to other protective effects, such as those acting on the cardiovascular system [10]. Moreover, Evodia is an important medicinal material used in a variety of prescriptions in TCM. However, its chemical composition is complex and includes many biologically active compounds that interact with multiple NPC-related therapeutic targets.

The article "Analysis of the Molecular Mechanism of Evodia rutaecarpa Fruit in the Treatment of Nasopharyngeal Carcinoma Using Network Pharmacology and Molecular Docking" was retracted in 2023. Reasons: suspected computer-generated content; unreliable results or conclusions; concerns about the data; concerns about the results or conclusions.

With the rapid growth and diversification of biological and drug data, it is necessary to adopt more extensive analytical techniques in systems biology. Network pharmacology methods based on systems biology and multidirectional pharmacology may be helpful to understand the interactions of various active components and determine their mechanisms of action. Several synergistic compounds in TCM prescriptions or monomers have been screened in a high-throughput manner, and the network regulation and rules have been elucidated.

Developing an Evodia-based treatment model that affects multiple signalling pathways based on its variety of active compounds could provide new strategies for treating diseases with complex pathophysiologies and multiple targets. Network pharmacology methods based on systems biology and polypharmacology can help elucidate the interactions between various active compounds. The complete method uses a “disease-target-drug” interaction network to identify connections between the active compounds of a drug and the disease target and attempts to clarify the synergy between the compounds and their potential mechanisms. Therefore, this method could clarify the mechanism of action of Evodia for NPC.

Current research on Evodia mainly focuses on its application for the treatment of cardiovascular diseases and other non-tumour diseases; however, its applicability to tumours, particularly those related to NPC, requires urgent attention. Therefore, in this study, we used network pharmacology and molecular-docking studies to predict the therapeutic targets of Evodia and its possible mechanisms of action in treating NPC. We subsequently verified the results using transcriptomic analysis and experiments. These results can provide a reference for subsequent research and promote new strategies involving the use of Evodia as targeted therapy for NPC.

## 2. Materials and Methods

### 2.1. Screening of Active Pharmaceutical Compounds

We used the TCM Systems Pharmacology (TCMSP) database and analysis platform to retrieve the chemical composition of Evodia [11]. To obtain the biologically active Evodia compounds, the search results were screened using oral bioavailability (OB; ≥30%) and drug-likeness (DL; ≥0.18) as the restrictive conditions [12]. Potential Evodia targets were then collected through the TCMSP platform and standardized using the UniProt database [13].

### 2.2. Disease-Related Gene Mining

To obtain NPC targets, we used “nasopharyngeal carcinoma” as a keyword for searches of the following five databases: GeneCard, OMIM, PharmGkb, the therapeutic targets database, and DrugBank. We merged the search results, deleted duplicate items, and obtained all NPC-related target genes.

The article "Analysis of the Molecular Mechanism of Evodia rutaecarpa Fruit in the Treatment of Nasopharyngeal Carcinoma Using Network Pharmacology and Molecular Docking" was retracted in 2023. Reasons: suspected computer-generated content; unreliable results or conclusions; concerns about the data; concerns about the results or conclusions.

### 2.3. Predicting the Therapeutic Target Gene Set

We matched the target-prediction results of the effective active Evodia compounds with the search results of NPC-related target genes and then used the Venn R package to compile a Venn diagram comprising targets of the effective active Evodia compounds and NPC target genes. We extracted cross-target Evodia genes and NPC targets as a common gene set to determine potential Evodia compounds for the treatment of NPC and then analysed the results.

### 2.4. Constructing a Network of Active Compounds and Associated Disease Targets

The screening results for the active Evodia compounds were imported into Cytoscape along with the NPC target-screening results [14] to construct a network of active compounds and NPC targets. We then used Network Analyzer to analyse the topological properties of the network, including the degree, betweenness centrality, and closeness centrality.

The nodes in the network represent a protein target or active compound, and the edges represent the interaction between these biomolecules. A node's impact increases with the number of direct connections with other nodes. The centrality between nodes is a measurement of the shortest path between them, and the closeness centrality is defined as the reciprocal of the average value of the shortest distances between a node and all other nodes in the network. The larger the value, the greater the centrality of the node, which also relates to the speed at which a signal is transmitted from one node to another [15, 16]. The node degree indicates the number of nodes connected in the network. A node with high betweenness centrality (BC) and closeness centrality (CC) values plays a very important role in the network.

### 2.5. Construction of a Protein-Protein Interaction (PPI) Network and Core Gene Screening

A PPI is formed when two or more protein molecules form a complex through non-covalent bonds. PPIs and the resulting networks are crucial in most biological functions and processes [17]. The STRING database contains known and predicted PPIs, and each PPI is annotated with one or more “scores” that are not indicative of the strength or specificity of the interaction but which represent an indicator of confidence. Thus, the likelihood of STRING judging an interaction to be true is based on the available evidence. All scores are ranked from 0 to 1, with 1 representing the highest possible confidence. A score of 0.5 indicates that roughly every second interaction is erroneous (i.e., a false positive). Based on this, the common gene targets of Evodia and NPC were imported into the STRING database. Using the *Homo sapiens* species, a confidence level of 0.7, and hidden disconnected nodes in the network, we performed a PPI network analysis and downloaded the results in TSV format.

The article "Analysis of the Molecular Mechanism of Evodia rutaecarpa Fruit in the Treatment of Nasopharyngeal Carcinoma Using Network Pharmacology and Molecular Docking" was retracted in 2023. Reasons: suspected computer-generated content; unreliable results or conclusions; concerns about the data; concerns about the results or conclusions.

The file was then imported into Cytoscape to conduct topology analysis, and CytoNCA was employed to calculate the six parameters used to evaluate the topological properties of the nodes within the interaction network [18]. These included the following: “degree centrality” (DC), BC, CC, “eigenvector centrality” (EC), “network centrality” (NC), and “local average connectivity” (LAC). These six parameters were used to indicate the nature of the nodes and determine their significance in the network. A node with high DC, BC, CC, EC, NC, and LAC values was considered to play an important role in the network. According to the results of the topological properties of the PPI network, targets above the median were selected as core targets, and two screening tests were conducted. Therefore, the core targets in the network were obtained.

### 2.6. Gene Ontology (GO) Biological Functional Analysis and Kyoto Encyclopaedia of Genes and Genomes (KEGG) Pathway Enrichment Analysis

GO and KEGG pathway enrichment analyses were conducted to analyse the target genes. An absolute value of the logarithmic fold change (>0.5) was the criterion for judging the significance of differentially expressed genes [19, 20]. The GO enrichment analysis provides a framework to describe the function of gene products in all organisms and to identify the biological characteristics or transcriptome data of high-throughput genomes. It uses three categories: molecular function, biological process, and cellular component. The KEGG database provides mRNA-related biological pathways enriched according to a given set of data. These analyses were conducted using the clusterProfiler R package [21], and the ggplot2 R package was used to display the results.

### 2.7. Molecular Docking to Identify Interactions between Drug and Target Compounds

Target protein structures were obtained from the Research Collaboratory for Structural Bioinformatics (RCSB) Protein Data Bank (PDB), and the two-dimensional structures of the active Evodia compounds were obtained from the PubChem database [22]. ChemBio Draw 3D (PerkinElmer, Billerica, MA, USA) and Autodock (https://autodock.scripps.edu/) were used to optimize the structures of key compounds and targets, which were used to determine three-dimensional (3D) chemical structures and perform energy minimization and format conversion [23]. PyMol was used to evaluate the proteins, remove ligands and water molecules, and perform the structural adjustments. Docking was carried out using R software and Autodock VINA. The molecule with the lowest binding energy in the docking conformation was selected, and the binding effect was observed via matching the original ligand and the interaction between the molecules.

The article "Analysis of the Molecular Mechanism of Evodia rutaecarpa Fruit in the Treatment of Nasopharyngeal Carcinoma Using Network Pharmacology and Molecular Docking" was retracted in 2023. Reasons: suspected computer-generated content; unreliable results or conclusions; concerns about the data; concerns about the results or conclusions.

### 2.8. Differential Expression Analyses

Based on the high specificity of antibody binding to an antigen, immunohistochemistry can reveal the relative distribution and abundance of proteins. Immunohistochemical data were obtained from the Human Protein Atlas (HPA), and the expression of target genes in normal and cancer tissues was compared [24]. Transcriptome data of cancer-related genes were obtained from The Cancer Genome Atlas (TCGA), including data related to 44 normal samples and 502 cancer samples. Differential expression analysis was conducted to verify the differences between the expression of target genes in cancer and cancer-adjacent samples. Additionally, transcription data of cancer and cancer-adjacent tissues from the same patient were extracted and paired to conduct differential expression analysis.

### 2.9. In Vitro Experimental Evaluation

Different mass concentrations (5, 10, 20, 40, and 80 *μ*mol·L^−1^) of isorhamnetin and a positive control (cisplatin, 4 *μ*g·mL^−1^) were used to treat NPC CNE-2 cells. Cell Counting Kit-8 (CCK-8) assays were used to detect the proliferation of CNE-2 cells, and Annexin V-fluorescein isothiocyanate (FITC)/propidium iodide (PI) dual-fluorescence staining was employed to detect the apoptosis rate [25].

### 2.10. Statistical Analysis

R software (v.3.6.1) was used to conduct statistical analyses. Unpaired *t*-tests were used to compare two groups of normally distributed variables, and the statistical significance of the non-normally distributed variables was estimated using the Mann–Whitney *U* test (Wilcoxon rank-sum test). The experimental verification results were processed using SPSS software (v.26.0; IBM Corp., Armonk, NY, USA), and data were visualized using GraphPad Prism software (v.8.0; GraphPad Software, La Jolla, CA, USA). The false discovery rate (FDR) method was used to adjust the *P*-value for multiple comparisons, and statistical significance was set to *P* < 0.05 (FDR <0.05).

## 3. Results

### 3.1. Research Process

Figure 1 shows a flowchart describing the process used to determine the effective target genes of Evodia for treating NPC and the experiments conducted to verify the results. The data sources used in this process and the websites visited for data analyses are provided in Table S1.

### 3.2. Screening of Active Evodia Compounds

In the TCMSP database, 30 active Evodia compounds were selected via screening, where OB greater than 30% and DL greater than 0.18 were the restrictive conditions (Table S2). Together with the compound retrieval results, we identified 24 active compounds for subsequent experiments (including indoles, quinolone alkaloids, physalin, and volatile oils) where certain compounds, such as quercetin, have been confirmed to inhibit the growth of tumour cells [26].

The article "Analysis of the Molecular Mechanism of Evodia rutaecarpa Fruit in the Treatment of Nasopharyngeal Carcinoma Using Network Pharmacology and Molecular Docking" was retracted in 2023. Reasons: suspected computer-generated content; unreliable results or conclusions; concerns about the data; concerns about the results or conclusions.

Additionally, 495 Evodia targets were obtained from the TCMSP database. These genes were integrated through the UniProt database, and invalid and duplicate targets were deleted. In addition, 170 target genes associated with the effective active compounds were acquired (Table S3).

### 3.3. Construction of a Target Gene Set for NPC

By integrating information from the GeneCard, OMIM, PharmGkb, TTD, and DrugBank databases, we obtained 8,953 gene targets for NPC (Figure 2(a)). We mapped the 170 target genes associated with the effective active Evodia compounds to the 8,953 target genes for NPC, identifying 153 composite target genes (Figure 2(b) and Table S4).

### 3.4. Identification of Active Compounds in the Evodia-NPC-Target Interaction Network

We used Cytoscape software to draw a diagram of the active compounds in the Evodia-NPC-target interaction network. The docking results for the 24 active Evodia compounds and 153 NPC targets (Figure 2(c) and Table S5) resulted in a network of 177 nodes and 269 edges. The complex interactions between nodes indicated that individual target genes of NPC were associated with one or more active Evodia compounds, with multiple targets also corresponding to the same active compounds, suggesting that Evodia contains multiple compounds for multiple targets potentially related to NPC treatment. We identified quercetin, isorhamnetin, *β*-sitosterol, evodiamine, goshuyuamide, and rutaecarpine as the primary Evodia compounds associated with potential NPC targets.

### 3.5. Construction of a Target PPI Network

We then used STRING to process the NPC targets of Evodia compounds to construct a PPI network, resulting in a network of 127 nodes and 1,006 edges (Figure 3(a)). Scoring of the network in Cytoscape according to BC, CC, DC, EC, NC, and LAC parameters (Figure 3(b)) revealed that the thresholds for the first round of screening were DC greater than 12, EC greater than 0.042378277, LAC greater than 4, BC greater than 58.28259727, CC greater than 0.352941176, and NC greater than 4.8, with the results showing 33 nodes and 363 edges (Figure 3(c)). We then scored these nodes a second time, and the resulting thresholds for the second round of screening were DC greater than 20, EC greater than 0.148225084, LAC greater than 9.142857143, BC greater than 14.7986531, CC greater than 0.581818182, and NC greater than 10.29488406. These results revealed 13 nodes and 120 edges (Figure 3(d) and Table S6), including retinoblastoma 1 (RB1), c-Jun N-terminal kinase (JUN), mitogen-activated protein kinase (MAPK) 14, cyclin D1, AKT1, heat shock protein 90 alpha family class A member 1, oestrogen receptor 1, MAPK1, MYC, hypoxia-inducible factor 1A, REL-associated protein (RELA), FOS, and p53. Therefore, these proteins were identified as the main potential therapeutic targets for treating NPC.

The article "Analysis of the Molecular Mechanism of Evodia rutaecarpa Fruit in the Treatment of Nasopharyngeal Carcinoma Using Network Pharmacology and Molecular Docking" was retracted in 2023. Reasons: suspected computer-generated content; unreliable results or conclusions; concerns about the data; concerns about the results or conclusions.

### 3.6. Biological Functional GO Analysis and Core Pathway Screening for Evodia in the Treatment of NPC

We used the Bioconductor R software package to conduct GO enrichment analysis of key targets. The screening was performed using a threshold of *P* < 0.05 (*Q* < 0.05), resulting in the identification of 2,118, 56, and 181 GO targets related to biological processes, cellular components, and molecular functions, respectively. The biological processes included responses to drugs, generation of reactive oxygen species (ROS), cellular response to chemical stress, response to lipopolysaccharides, and response to molecules of a bacterial origin. The top 20 GO terms are displayed in Figures 4(a) and 4(b) and in Table S7.

KEGG enrichment analysis of the 153 Evodia targets showed that they were enriched in 177 signalling pathways, including those related to hepatitis B, fluid shear stress and atherosclerosis, chemical carcinogenesis-receptor activation, and lipid and atherosclerosis, each of which play important roles in NPC development and progression. We displayed the top 20 KEGG enrichment results in Figures 4(c) and 4(d) and in Table S8. Notably, pathways associated with lipids and atherosclerosis were the most highly enriched signalling pathways (Figure 5). The GO and KEGG results showed that Evodia compounds potentially act on multiple NPC-specific pathways.

### 3.7. Molecular Docking Studies to Evaluate Interactions between Active Evodia Compounds and NPC Targets

Based on the KEGG enrichment analysis, the top six target proteins in the PPI network and their corresponding active compounds were selected for molecular docking. Data for the following proteins were downloaded from the PDB: MAPK14 (PDB ID: 2RG6), AKT1 (PDB ID: 7NH5), RELA (PDB ID: 5URN), JUN (PDB ID: 5T01), MAPK1 (PDB ID: 7NR9), and p53 (PDB ID: TBWN). Docking of the 3D structures with their respective compounds was visualized using PyMol, with lower binding energy designating a high-affinity interaction (Figure 6). The binding energy values of most Evodia compounds were below −1 kcal∙mol^−1^, indicating that they possessed good binding activity. The results identified hydrogen bonding and *π*-*π*-stacking interactions, which suggested potential favourable interactions between the compounds and NPC targets.

The article "Analysis of the Molecular Mechanism of Evodia rutaecarpa Fruit in the Treatment of Nasopharyngeal Carcinoma Using Network Pharmacology and Molecular Docking" was retracted in 2023. Reasons: suspected computer-generated content; unreliable results or conclusions; concerns about the data; concerns about the results or conclusions.

### 3.8. Differential Expression of Target Genes in NPC

To verify the potential of the identified proteins as therapeutic targets, we analysed the differential expression of proteins in NPC tissues and cancer-adjacent tissues. Immunohistochemical results from the HPA database showed that JUN expression in cancer tissues was higher than that in normal nasopharyngeal tissues, whereas antibody staining levels of MAPK14, AKT1, and MAPK1 in cancer tissues were lower than those in adjacent tissues. However, we observed no significant differences in RELA and p53 expression between tumour and normal nasopharyngeal tissues (Figure 7(a)).

We used the TCGA database to expand the sample size for verification and obtain more accurate results. The box plot of the differential expression analysis (Figure 7(b)) showed that the expression of MAPK14, MAPK1, AKT1, and RELA was significantly higher in cancer tissues than in normal tissues. Furthermore, the paired analysis identified significantly higher MAPK1, AKT1, and RELA expression in cancer tissues than in cancer-adjacent tissues from the same patient (Figure 7(c)).

### 3.9. Experimental Verification

Based on previous reports and preexperimental results, we selected isorhamnetin for experimental verification of its influence on the biological processes of NPC cell proliferation and apoptosis. CCK-8 assays showed that treatment of CNE-2 cells with isorhamnetin (5, 10, 20, 40, and 80 *μ*mol·L^−1^) for 24, 36, and 48 h significantly inhibited cell proliferation compared with cisplatin treatment (4 *μ*g·mL^−1^; *P* < 0.05; Figure 8(a)). Additionally, Annexin V-FITC/PI dual-fluorescence staining showed that isorhamnetin increased the apoptosis rate of NPC cells at 48 h (Figure 8(b)). These findings indicated that isorhamnetin induced NPC cell apoptosis.

## 4. Discussion

Given the increase in the prevalence of individualized diagnosis and treatment of disease, NPC morbidity and mortality have decreased to varying degrees in recent decades [27]. Preventing adverse reactions caused by individualized chemotherapy and intensity-modulated radiotherapy and increasing the clinical benefits to patients can positively impact the clinical success rate of NPC treatment. Numerous studies on NPC prevention and treatment have been conducted to identify new and effective treatment strategies that are less toxic and have fewer adverse effects than current regimens. In this respect, providing an individualized diagnosis and treatment regimen supplemented with natural products and their derivatives would be beneficial for treating NPC. TCM provides a more holistic approach to the diagnosis and treatment of tumours than Western medicine; the main pathogenesis of NPC is believed to be a deficiency of righteous qi, an internal accumulation of heat toxin, and intermingled phlegm and blood stasis. Of these, qi-deficiency-induced toxin contamination is regarded as the most important cause of NPC.

The article "Analysis of the Molecular Mechanism of Evodia rutaecarpa Fruit in the Treatment of Nasopharyngeal Carcinoma Using Network Pharmacology and Molecular Docking" was retracted in 2023. Reasons: suspected computer-generated content; unreliable results or conclusions; concerns about the data; concerns about the results or conclusions.

Evodia is recorded in ancient medicine books and has a long history of medicinal use. Modern pharmacological studies have shown that Evodia has analgesic [28], anti-inflammatory [29], anti-bacterial [30], anti-emetic, anti-diarrheal, and anti-tumour [31] properties, and biochemical analyses have demonstrated that Evodia mainly contains the following compounds: alkaloids, bitterin, volatile oil, and flavonoids. Of these, the most effective active compounds are reportedly quercetin, isorhamnetin, *β*-sitosterol, evodiamine, goshuyuamide, and rutaecarpine.

Previous studies have suggested that several active Evodia compounds exert cytotoxic effects on human cancer cell lines. Specifically, evodiamine has inhibitory effects on A549 human lung cancer cells [32], and limonin in Evodia induces apoptosis in ovarian cancer cells by activating the p53 signalling pathway [33]. Additionally, evodiamine plays an important role in activating c-Jun N-terminal kinase (JNK) and protein kinase R-like endoplasmic reticulum kinase (PERK) in human ovarian cancer cells to induce apoptosis [34] and inhibits the proliferation of hepatocarcinoma cells through a WW domain containing oxidoreductase-dependent pathway to induce anti-cancer activity [35]. Moreover, evodiamine may induce bladder cancer cell apoptosis through mammalian target of rapamycin (mTOR)/S6 kinase 1-mediated myeloid cell leukaemia-1 downregulation and enhance tumour necrosis factor-related apoptosis-inducing ligand-induced apoptosis [36]. These findings suggest the potential efficacy of Evodia in anti-tumour treatment.

However, Evodia displays a certain degree of hepatotoxicity, and adverse events have been reported in clinical practice. Therefore, exploring the specific Evodia compounds effective for tumour treatment, as well as their respective mechanisms of action, will help develop and promote their safe future use. Molecular docking is a computer analysis technology based on structures and ligands that is widely used to elucidate how compounds interact with their molecular targets in drug discovery and development. We searched for therapeutic compounds by reverse screening the ligands of the protein structure library and evaluating their binding affinity. This necessitates further research on possible NPC targets of Evodia compounds.

The article "Analysis of the Molecular Mechanism of Evodia rutaecarpa Fruit in the Treatment of Nasopharyngeal Carcinoma Using Network Pharmacology and Molecular Docking" was retracted in 2023. Reasons: suspected computer-generated content; unreliable results or conclusions; concerns about the data; concerns about the results or conclusions.

In this study, 24 active Evodia compounds and 153 NPC targets were used to construct a target interaction network, and the results showed that most Evodia compounds affected multiple NPC targets. Specifically, quercetin, isorhamnetin, evodiamine, and *β*-sitosterol interacted with 121, 26, 26, and 25 targets, respectively, suggesting that they may act as pleiotropic compounds. Although each compound showed interactions with multiple targets, many of these target-compound interactions overlapped, suggesting a possible synergistic effect between the compounds.

Quercetin is found in many fruits and vegetables, and many studies have investigated the molecular mechanisms of quercetin in NPC treatment. For example, a previous report confirmed that quercetin exerts anti-cancer effects on a variety of tumour cells by regulating the phosphatidylinositol 3-kinase (PI3K)/Akt/mTOR, Wnt/*β*-catenin, and MAPK/extracellular signal-regulated kinase 1/2 signalling pathways [26]. Additionally, quercetin inhibits angiogenesis in NPC tumours [37] and induces growth inhibition and apoptosis of NPC cells [38, 39]. Furthermore, quercetin is used in cisplatin combination chemotherapy, where it exerts a significant synergistic effect.

Isorhamnetin is a representative flavonoid compound that exhibits anti-tumour activity primarily by inhibiting tumour cell proliferation, inducing apoptosis, and inhibiting signal transduction. For example, Cai et al. reported that isorhamnetin inhibits the proliferation and metastasis of androgen-independent prostate cancer cells by targeting the endogenous apoptotic pathway and selectively inhibiting PI3K/AKT/mTOR signalling [40].

Natural products are highly complex, and their effects on the treatment of diseases may result from the combined action of multiple compounds. Our results showed that quercetin, evodiamine, and isorhamnetin were associated with many NPC targets. GO enrichment analysis showed that NPC targets of Evodia compounds were involved in biological processes related to NPC development, including drug response, generation of ROS, and cellular response to chemical stress. Furthermore, Chaaben et al. reported that dysfunctional gene-driven redox stress pathways may increase the risk of disease in NPC-susceptible individuals [41].

Uncontrolled tumour cell proliferation is related to abnormal gene expression and signal transduction. The current findings suggested that Evodia may interfere with these pathological processes to inhibit NPC cell proliferation and promote their apoptosis. Our KEGG pathway analysis showed that Evodia compounds affect NPC via multiple signalling pathways that overlap with lipid- and atherosclerosis-related signalling pathways. Analysis of these signalling pathways revealed 37 common biomarkers, including lectin-like oxidized low-density lipoprotein receptor-1 (LOX-1), AKT, nuclear factor (NF) *κ*B, and p53, which are important in cell proliferation, apoptosis, migration, and invasion. A previous study showed that LOX-1 alters ROS production, leading to lipid peroxidation and DNA damage, and promotes atherosclerosis and cancer progression, suggesting that LOX-1 inhibition may be a promising therapeutic strategy [42]. Therefore, these biomarkers could represent a potential link between atherosclerosis and cancer and provide insight into the associated molecular mechanisms.

The article "Analysis of the Molecular Mechanism of Evodia rutaecarpa Fruit in the Treatment of Nasopharyngeal Carcinoma Using Network Pharmacology and Molecular Docking" was retracted in 2023. Reasons: suspected computer-generated content; unreliable results or conclusions; concerns about the data; concerns about the results or conclusions.

The generated PPI network identified six targets for molecular docking studies, namely MAPK14, AKT1, RELA, JUN, MAPK1, and p53. AKT1 is a key regulator of PI3K/AKT signalling and participates in cell proliferation and apoptosis [43]. MAPK14 and MAPK1 are important members of the MAPK family, and MAPK14 is an important biomarker of metastatic gastric cancer, where its inhibition significantly reduces the progression of advanced gastric cancer [44]. Additionally, MAPK1 affects the progression of breast and ovarian cancers by participating in multiple signalling pathways [45, 46], and AKT1 is closely related to cancer and a variety of diseases through its roles in metabolic regulation and signalling pathways [47, 48]. *RELA* is an important target gene in NF-*κ*B signalling; Lu and Yarbrough [49] reported that *RELA* dephosphorylation inhibits tumour development [49], and other studies have indicated that *RELA* methylation and subsequent activation of multiple downstream genes contribute to the regulation of breast cancer progression [50, 51]. JUN is an activator protein-1 transcription factor subunit that regulates the expression of multiple genes critical to cell proliferation, differentiation, and apoptosis [52]. TP53 is the most commonly mutated tumour suppressor gene in human cancers, with its mutations closely related to a variety of cancers, and it is being targeted for the development of numerous treatment strategies [53].

## 5. Conclusion

As a TCM, *E. rutaecarpa* has achieved remarkable results in clinical practice and is an important component in the combination therapy of NPC with other drugs. Reports on the mechanisms of action of natural plants in the treatment of NPC are scarce; therefore, this study offers new insights into the study of Evodia and its applications as adjuvant therapy. Elucidation of the mechanisms through which *E. rutaecarpa* exerts curative effects will be beneficial. In this study, we identified the effective active components of Evodia and target molecules in NPC. Our findings suggested that continued evaluation of evodiamine and other active components is warranted for their possible application in treating NPC and for supporting the scientific basis of using natural plants to treat NPC.

The article "Analysis of the Molecular Mechanism of Evodia rutaecarpa Fruit in the Treatment of Nasopharyngeal Carcinoma Using Network Pharmacology and Molecular Docking" was retracted in 2023. Reasons: suspected computer-generated content; unreliable results or conclusions; concerns about the data; concerns about the results or conclusions.

## Figures and Tables

**Figure 1:** Flow diagram of the systematic analysis and validation processes.

**Figure 2:** Construction of the target gene set and compound-target network: (a) Venn diagram of NPC target genes from the GeneCard, OMIM, PharmGkb, TTD, and DrugBank databases; (b) Venn diagram of Evodia compounds and NPC targets; and (c) Evodia compound;target network. The red rectangular nodes are the main active Evodia compounds, and the blue rectangle is the potential NPC target for treatment using the Evodia compounds.

**Figure 3:** Generated PPI network: (a) PPI network of NPC targets of Evodia compounds; (b) PPI network containing 127 nodes and 1,006 edges where areas highlighted in yellow represent the candidate targets ranked according to median values of DC, BC, CC, EC, LAC, and NC; (c) PPI network containing 33 nodes and 363 edges where areas highlighted in yellow represent potential targets with median values of DC, BC, CC, EC, LAC, and NC; and (d) PPI network containing 13 potential targets with median values for DC, BC, CC, EC, LAC, and NC.

**Figure 4:** Top 20 GO-enriched terms and KEGG pathway annotations. (a, b) GO enrichment of active Evodia compounds for application against NPC targets. (c, d) Enriched KEGG pathways of potential NPC targets using active Evodia compounds.

**Figure 5:** Pathway map of Evodia compounds for their potential treatment of NPC. NPC targets related to the Evodia compounds are involved in “lipid and atherosclerosis” pathways. Arrows represent activation; T-arrows represent inhibition; and segments show either activation or inhibition.

**Figure 6:** Molecular docking of Evodia compounds with NPC targets.

**Figure 7:** Differential expression of NPC targets: (a) validation of the expression of NPC targets at the protein level using the HPA database (immunohistochemistry), (b) differential expression of NPC targets, and (c) paired difference analysis of NPC targets.

**Figure 8:** Experimental verification: (a) isorhamnetin inhibits the proliferation of CNE2 cells according to the CCK-8 assay ($\bar{X}\pm s,n=3$) and (b) isorhamnetin promotes CNE2 cell apoptosis ($\bar{X}\pm s,n=3$).

## Data Availability

The data sets used in this paper are available from the corresponding author upon request.

## Abbreviations

NPC: Nasopharyngeal carcinoma
GO: Gene ontology
KEGG: Kyoto Encyclopaedia of Genes and Genomes
TCGA: The Cancer Genome Atlas
HPA: Human Protein Atlas
EBV: Epstein–Barr virus
TCM: Traditional Chinese medicine
TCMSP: TCM systems pharmacology
OB: Oral bioavailability
DL: Drug-likeness
BC: Betweenness centrality
CC: Closeness centrality
PPI: Protein-protein interaction
DC: Degree centrality
EC: Eigenvector centrality
NC: Network centrality
LAC: Local average connectivity.

The article "Analysis of the Molecular Mechanism of Evodia rutaecarpa Fruit in the Treatment of Nasopharyngeal Carcinoma Using Network Pharmacology and Molecular Docking" was retracted in 2023. Reasons: suspected computer-generated content; unreliable results or conclusions; concerns about the data; concerns about the results or conclusions.

## Supplementary Materials

Supplementary Materials Table S1: database and website. Table S2: active ingredient parameters of ER. Table S3: potential target information of ER. Table S4: common gene of ER in the treatment of NPC. Table S5: ER active ingredients and NPC target network. Table S6: core gene of PPI network. Table S7: the data of GO enrichment analysis. Table S8: the data of KEGG pathway enrichment analysis.
